# Extreme Learning Machine for Heartbeat Classification with Hybrid Time-Domain and Wavelet Time-Frequency Features

**DOI:** 10.1155/2021/6674695

**Published:** 2021-01-11

**Authors:** Yuefan Xu, Sen Zhang, Zhengtao Cao, Qinqin Chen, Wendong Xiao

**Affiliations:** ^1^School of Automation & Electrical Engineering, University of Science and Technology Beijing, Beijing 100083, China; ^2^Air Force Medical Center,PLA, Beijing 100142, China; ^3^China Academic of Electronics and Information Technology of CETC, Beijing 100041, China; ^4^Beijing Engineering Research Center of Industrial Spectrum Imaging, Beijing 100083, China

## Abstract

Automatic heartbeat classification via electrocardiogram (ECG) can help diagnose and prevent cardiovascular diseases in time. Many classification approaches have been proposed for heartbeat classification, based on feature extraction. However, the existing approaches face the challenges of high feature dimensions and slow recognition speeds. In this paper, we propose an efficient extreme learning machine (ELM) approach for heartbeat classification with multiple classes, based on the hybrid time-domain and wavelet time-frequency features. The proposed approach contains two sequential modules: (1) feature extraction of heartbeat signals, including RR interval features in the time-domain and wavelet time-frequency features, and (2) heartbeat classification using ELM based on the extracted features. RR interval features are calculated to reflect the dynamic characteristics of heartbeat signals. Discrete wavelet transform (DWT) is used to decompose the heartbeat signals and extract the time-frequency features of the heartbeat signals along the timeline. ELM is a single-hidden layer feedforward neural network with the hidden layer parameters randomly generated in advance and the output layer parameters calculated optimally using the least-square algorithm directly using the training samples. ELM is used as the heartbeat classification algorithm due to its high accuracy training accuracy, fast training speed, and good generalization ability. Experimental testing is carried out using the public MIT-BIH arrhythmia dataset to perform a 16-class classification. Experimental results show that the proposed approach achieves a superior classification accuracy with fast training and recognition speeds, compared with existing classification algorithms.

## 1. Introduction

Arrhythmia is caused by disturbance in the rate, regularity, site of origin, or conduction of the cardiac electrical impulse [1]. Severe arrhythmias can even threaten human life. An electrocardiogram (ECG) records the changes in electrical activity generated during each cardiac cycle of the heart, which can help doctors to diagnose arrhythmias. However, a routine ECG usually lasts only a few minutes, which sometimes does not detect an occasionally irregular heart rhythm. Some cardiovascular diseases, such as sudden cardiac death caused by ventricular tachyarrhythmia, have short durations from onset to death. The Holter monitor, a portable device invented by Norman J. Holter in 1949, can continuously monitor the patient's electrical activity of the heart for 24 hours or more in their daily life [2]. The extended monitoring period is helpful to observe occasional cardiac arrhythmias which would be difficult to be detected in a shorter period. Besides, due to the numerous varieties and subtle changes of heartbeats, usually arrhythmia needs to be identified by experienced doctors. The automatic arrhythmia classification approach based on ambulatory ECG plays a role in timely detecting arrhythmia and therefore can effectively prevent the cardiovascular diseases.

Two main factors affect the performance of heartbeat classification: features extracted from the heartbeat signals, and selected classifier. The extracted features should show dispersions between different heartbeat types and the similarities between features within the same heartbeat type. In the literature, various handcrafted features have been extracted for heartbeat classification, including RR interval features [3, 4], morphological features [5], wavelet features [6, 7], independent component analysis [8], and higher-order statistics [9]. Recent studies tend to automatically extract the features of heartbeat signals via deep learning [10–12].

For classification task, classifiers such as support vector machine (SVM) [13], k-nearest neighbor (KNN) [14], and backpropagation neural network (BPNN) [15] have been used. However, the training speed of gradient descent based BPNN is slow, and its parameters often fall into local optimums. For SVM, the training time increases exponentially as the feature dimension increases. Faced with so many features, feature reduction is often performed first, followed by classification. Extreme learning machine (ELM) is originally developed for the single-hidden layer feedforward neural networks (SLFNs), and then extended to the generalized SLFNs which need not be neuron alike [16]. The hidden layer parameters are randomly generated, and the output parameters are calculated analytically. ELM is iteration-free, so its training speed is very fast compared with the BPNN algorithm. Huang et al. prove that ELM has universal approximation capability [17]; that is, as the number of hidden layer nodes increases, the network can approximate nonlinear functions with infinitely small errors.

Due to these advantages, ELM has been studied extensively over the years, and many different types of ELM have been proposed to solve different machine learning problems. Liang et al. [18] proposed an online sequential ELM (OS-ELM) which is used in the situation that the training samples are processed one by one. Zong et al. [19] proposed the weighted ELM (W-ELM) when the numbers of samples of different classes are imbalanced. Huang et al. [20] extended ELM using kernel trick (KELM), which greatly improves the performance of ELM, and they explained why ELM is the optimal solution, while SVM is the suboptimal solution. The experimental results also verified that the performance of KELM is better than SVM. To make full use of unlabeled samples, semisupervised ELM (SS-ELM) and unsupervised ELM (US-ELM) were proposed [21]. Tang et al. [22] designed a multilayer ELM (ML-ELM) in which feature extraction and classification are integrated into a unified network structure. The multilayer structure of ML-ELM increases the representation ability of ELM, which can extract features automatically. Zhang et al. [23] proposed residual compensation ELM (RC-ELM) for regression problem, which employs a multilayer structure. The residual is compensated layer by layer iteratively by remodeling the unmodeling prediction error in the previous layer. Recently, they [24] proposed a robust ELM (R-ELM) to improve the modeling capability and robustness with unknown noise. They used mixture of Gaussian to fit the noise and constructed a modified objective function.

In this paper, we will propose an efficient ELM approach for heartbeat classification with multiple classes based on the hybrid time-domain and wavelet time-frequency features. We extract the RR interval features in time-domain and wavelet time-frequency coefficient features of the heartbeats. Four types of RR intervals are calculated to reflect the temporal characters of heartbeat signals. Discrete wavelet transform (DWT) is employed to decompose the heartbeat signal to wavelet coefficient components that progress over time, and wavelet decomposition coefficients are designated as the time-frequency features. We concatenate these two types of features, forming a total of 20 heartbeat features. Then, ELM is introduced to classify the heartbeat signals into 16 categories.

The main contributions of this paper include the following: (1) temporal features and time-frequency features are simultaneously extracted for heartbeat signals. The integrated features capture the characteristics of heartbeat signals more comprehensively; (2) ELM is introduced to achieve high heartbeat classification accuracy and recognition speed.

The paper is organized as follows: Section 2 presents the related work.  Section 3 briefly introduces ELM.  Section 4 details the feature extraction schemes and the proposed approach.  Section 5 reports the experimental results. Finally, Section 6 presents the conclusions and the future work.

## 2. Related Work

In the literature, feature extraction methods for heartbeat signals can be mainly classified to two categories: manually feature extraction and automatically feature extraction. For the former, handcrafted features will reflect meaningful information for original ECG signals in specific aspects. Recently, with the popularity of deep learning, scholars begin to design neural networks with deep structures that are suitable for ECG signals and automatically extract the features in a layer-by-layer manner.

Khalaf et al. [25] introduced cyclostationary signal analysis to extract heartbeat features. They used the spectral correlation as a nonlinear statistical transformation to inspect the periodicity of the correlation. However, the large number of features was extracted by this method, and the author employed principal component analysis (PCA) to reduce the feature dimensions. Finally, SVM classifies the heartbeat signals into 5 categories. Mert [26] decomposed electrocardiogram beats into a set of band-limited oscillations by variational mode decomposition (VMD). The amplitude modulation bandwidth, the frequency modulation bandwidth, and the total bandwidth of the modes form the feature vectors. Then, the bagged decision tree is adopted to classify the heartbeat into six classes.

Ye et al. [13] extracted dynamic and morphological features of the heartbeat signal. A total of 128 features are obtained, which consist of 114 wavelet features and 14 independent component coefficient features. Then, PCA is used to reduce the feature dimensions, and SVM for classification. The process of extracting so many features and then reducing dimensionality is redundant when classifying the heartbeat signals. The introduction of PCA may lose the original information.

Wavelet transform (WT) has been developed for automatic ECG analysis, including signal denoising, wave detection, and heartbeat classification [27]. Li et al. [28] employed DWT with soft thresholding to reduce the noises of the ECG signals. Biswas et al. [29] gave the detailed comparisons of different wavelet families on ECG denoising. Kaur et al. [30] detected the QRS complexes by DWT with Db6 wavelet. By the convolution operation of the wavelet basis function and the ECG signals, the peak can be found at the position corresponding to the largest convolution result, due to the morphological similarity between wavelet and QRS complexes. Sarkaleh and Shahbahrami [15] calculated the statistics of the DWT coefficients and selected BPNN as the classifier. When WT is acted as a feature extractor, it can actually be regarded as a downsampling operation.

Recently, Yildirim et al. [10] proposed to automatically extract heartbeat features via deep learning methods. They designed a convolutional autoencoder to reduce the signal size of arrhythmic beats. Then, long short-term memory (LSTM) classifiers were employed to automatically recognize heartbeat classes. Fan et al. [31] proposed a multiscaled fusion of the deep convolutional neural network to recognize atrial fibrillation. Two-stream convolutional networks with different filter sizes were customized to capture features of different scales. Although this method can automatically extract features, the deep learning-based feature extraction method is black-box and cannot effectively explain the meaning of the extracted features.

ELM has been applied to many applications. Mohammed et al. [32] employed ELM for face recognition, producing a faster recognition rate. Yuan et al. [33] classified epilepsy patients via EEG, and ELM was chosen as the classifier. Experimental results demonstrated satisfactory classification accuracy and fast training time. Huang et al. [34] used ELM to recognize traffic signs. The proposed method not only has a high recognition rate but also has high computational efficiency in both training and recognition process. Zhang et al. [35] performed parameterized geometrical feature extraction (PGFE) and designed an ELM-based approach for device-free localization, which can improve the localization accuracy significantly. Later, they continued to develop ELM and applied it to large-scale device-free localization setting, and experimental results showed the validity of the proposed approach [36]. However, less work involves the use of ELM to classify heartbeat signals, and ELM is not fully developed to perform multiclass heartbeat classification.

Kim et al. [6] extracted the heartbeat features by continuous wavelet transform, and ELM was carried out for classification. However, ELM without constraints on output parameters of SLFN tends to perform poorly.

## 3. Extreme Learning Machine

ELM is a single-hidden layer feedforward neural network, which contains three layers, namely, the input layer, the hidden layer, and the output layer.  Figure 1 shows the structure of ELM. The parameters in ELM are calculated in a different way from BP. The hidden layer parameters are randomly generated, and the output parameters connecting the hidden layer and the output layer are analytically obtained by the least-square method.

ELM has the universal approximation ability [17]. Specifically, given any bounded nonconstant piecewise continuous activation function, a network with randomly generated hidden layer parameters can approximate the objective function with an arbitrarily small error, simply by adjusting the output parameters.

Now, we briefly present the principle of ELM.

Suppose that we have *N* labeled samples *x*_*i*_, where *i*=1,2,…, *N* and *x*_*i*_ ∈ *R*^*n*^. The parameters of the hidden neurons are randomly generated according to any continuous probability distribution; then, for SLFNs with *L* hidden neurons, the hidden layer output matrix *H* is calculated forward as

(1) $$\begin{array}{c} H={\left[\begin{array}{ccc} g\left(a_{1}\cdot x_{1}+b_{1}\right) & \cdots & g\left(a_{L}\cdot x_{1}+b_{L}\right)\\ \vdots & \vdots & \vdots \\ g\left(a_{1}\cdot x_{N}+b_{1}\right) & \cdots & g\left(a_{L}\cdot x_{N}+b_{L}\right) \end{array}\right]}_{N\times L}, \end{array}$$

where *g*(·) is the activation function and *a*_*i*_ and *b*_*i*_ are the parameters of the *i*th hidden node in the hidden layer. The propagation of data from the input layer to the hidden layer actually maps the original data from the *n*-dimensional space to the *L*-dimensional space.

For multiclass classification, the number of ELM output nodes is set to the same as the number of the classes. Assuming that there are *m* classes, *c* is the original class label, and the expected output vector of the *m* output nodes is encoded as $t_{i}={\left[-1,\ldots ,-1,\overset{c}{1},-1,\ldots ,-1\right]}^{T}$; that is, only the *c*th element of *t*_*i*_ is 1, while the rest elements are set to −1. The relationship between the output of the hidden layer and the network is written as

(2) $$\begin{array}{c} H\beta =T, \end{array}$$

where

(3) $$\begin{array}{c} \beta ={\left[\begin{array}{ccc} \beta_{11} & \cdots & \beta_{1m}\\ \vdots & \ddots & \vdots \\ \beta_{L1} & \cdots & \beta_{Lm} \end{array}\right]}_{L\times m}, \end{array}$$

(4) $$\begin{array}{c} T={\left[\begin{array}{ccc} t_{11} & \cdots & t_{1m}\\ \vdots & \ddots & \vdots \\ t_{N1} & \cdots & t_{Nm} \end{array}\right]}_{N\times m}. \end{array}$$

Often the number of training samples is not equal to the number of hidden nodes; that is, the hidden layer output matrix *H* is not a square matrix, so the least-square solution of (2) is not unique. Bartlett pointed out that for feedforward neural network, the smaller the network weights, the better the generalization performance of the network [41]. The smallest norm least-square solution of *β* is

(5) $$\begin{array}{c} \hat{\beta }={Η}^{†}T, \end{array}$$

where Η^†^ is the Moore–Penrose generalized inverse of Η.

To avoid ill-posed problem, a positive value *C* is added to the diagonal of Η^*T*^Η according to the ridge regression theory. Then, the objective function of regularized ELM becomes

(6) $$\begin{array}{c} \text{Minimize}:l=\frac{1}{2}{\left\|\beta \right\|}^{2}+\frac{1}{2}C{\left\|T-H\beta \right\|}^{2}. \end{array}$$

Taking the derivative with respect to *β* and letting it be zero, then the output parameters of ELM are

(7) $$\begin{array}{c} \beta ={\left(\frac{Ι}{C}+H^{T}H\right)}^{-1}H^{T}T, \end{array}$$

where *I* is the unit matrix.

We summarize ELM into three steps, which are presented as follows:

1. Randomly generate the hidden layer parameters *a*_*i*_ and *b*_*i*_ according to any continuous probability distribution
2. Calculate the output matrix *H* of the hidden layer
3. Obtain the output parameters using equation (7)

## 4. Proposed Approach

In this section, we first introduce the MIT-BIH arrhythmia dataset and then detail the proposed heartbeat classification approach.

### 4.1. Dataset

The MIT-BIH arrhythmia dataset is one of the widely used datasets for the study of arrhythmia classification [37]. It contains 48 half-hour records of dual-channel dynamic ECG, which are obtained from 47 subjects. In these records, 23 records are randomly selected from 4000 24-hour Holter ECG records and 25 records are selected from the same set to include less common but clinically significant arrhythmias [38].

In the upper channel, 45 records of the signals are collected from a modified limb lead II (MLII) and 3 records are collected from a modified precordial lead V5. In the lower channel, 1 record is collected from MLII and the others are collected from lead V1, V2, V4, or V5. In our study, we use the signals of the upper channel and reverse two channels of record 114 to ensure that the signal comes from MLII.

All records are band-pass filtered at the range of 0.1–100 Hz, and then the filtered signals are digitized at 360 Hz. The dataset provides the label of each heartbeat, which is annotated by two cardiologists. The approximate location of the fiducial *R* point of each heartbeat is also marked in the dataset.

Table 1 gives the name, abbreviation, and annotation of each heartbeat type in the MIT-BIH arrhythmia dataset.

### 4.2. The Overall Structure

Figure 2 shows the overall structure of the proposed heartbeat classification approach. It contains two phases: the offline training phase and the online classification phase. Both phases consist of three stages, namely, preprocessing, heartbeat segmentation, and hybrid feature extraction. In the preprocessing stage, we eliminate the baseline wander of the ECG signals using median filters. Then, we divide the continuous heartbeat signal to heartbeat segments one by one. Next, we extract the RR interval features and wavelet coefficient features of the heartbeat signals. ELM is trained on the offline heartbeat training data, and finally, the trained ELM model classifies the online heartbeat signals.

### 4.3. Preprocessing

The baseline wander of ECG signal is caused by low-frequency interferences such as the respiration of the measured object and electrode movement. ECG signal contains low-frequency components, and the baseline wander will obscure useful information. Awodeyi et al. [39] proposed a novel approach for removal of baseline wander in photoplethysmography signals. We refer to this approach and design a two-stage median filtering approach to remove the baseline wander of ECG signal.

### 4.4. Heartbeat Segmentation

Before feature extraction, continuous ECG signal should be divided into individual heartbeats. A heartbeat segment should capture the useful information of the current heartbeat as much as possible, but avoid covering the components of the previous heartbeat or the next heartbeat.

Generally, the PR interval ranges from 0.12 to 0.22 seconds, and the QT interval is roughly less than 0.45 seconds, so without loss of generality, in this paper we set the duration of the heartbeat segmentation as 0.65 seconds. The MIT-BIH arrhythmia dataset provides the approximate location of the fiducial *R* point for each heartbeat. We manually correct the provided *R*-peak positions beat-by-beat. Then, based on the position of the corrected fiducial *R* point, the intervals of 0.25 seconds before *R* peak and 0.4 seconds after *R* peak are selected and they constitute a heartbeat segment of 0.65 seconds.

### 4.5. Feature Extraction

#### 4.5.1. RR Interval Features in the Time Domain

RR interval can reflect the relationship between the current heartbeat and its neighboring heartbeat in the time domain. This sequential relationship can help more effectively distinguish heartbeat signals. We calculate 4 types of RR interval information: previous RR, the interval between the *R* peak of the current heartbeat and the previous heartbeat; post RR, the interval between the *R* peak of the current heartbeat and the next heartbeat; short-term RR, the average interval of *l* previous RRs; long-term RR, the average interval of previous RRs over the *d* minutes before the current heartbeat. In this paper, we empirically choose *l* as 10 and *d* as 5.

To illustrate the effectiveness of RR interval features, we choose three heartbeat classes, each of which contains 50 randomly selected samples, and then plot scatter diagrams of their distributions.  Figure 3(a) shows that heartbeat classes atrial premature contraction (A), nodal (junctional) premature beat (J), and paced beat (/) can be easily distinguished by the feature of previous RR. From Figure 3(b), we can also find that heartbeat classes fusion of ventricular and normal beat (F), ventricular flutter wave (!), and blocked atrial premature beat (x) are clearly distinguished by the feature of long-term RR.

#### 4.5.2. Wavelet Time-Frequency Features

ECG signal is nonstationary signal; that is, its frequency changes over time. Using Fourier transform, we can only get the frequency components in the signal, but the specific time when these frequencies occur is not known. Although short-time Fourier transform (STFT) solves the above problem by adding a sliding window, it also faces the challenge that the window size is difficult to determine. Wavelet transform (WT) is a novel transform analysis method, which inherits and develops the idea of localization of STFT, and overcomes the shortcoming of STFT which the window size not changes with frequency. Below we first briefly introduce the definition of WT and then propose the wavelet coefficient features of heartbeat signals extracted by WT.

WT uses multiple changeable “time-frequency” windows and provides the localized analysis of time and frequency. By gradually refining the signal in multiple scales through extension and translation operations, WT finally achieves time subdivision at high frequency and frequency subdivision at low frequency, which makes it an ideal tool for signal time-frequency analysis and processing.

WT is divided into continuous WT (CWT) and discrete WT (DWT). Formally, CWT is described as

(8) $$\begin{array}{c} X\left(a,\tau \right)=\frac{1}{{\left|a\right|}^{1/2}}\int_{-\infty }^{\infty }x\left(t\right)\bar{\psi }\left(\frac{t-\tau }{a}\right)\text{d}t, \end{array}$$

where *x*(*t*) is the given signal, *ψ*(*t*) is continuous mother wavelet, *a* is the scaling parameter, and *τ* is the translating parameter, and their values are continuous, which means the number of wavelets is unlimited. Wavelet can be scaled by scaling parameter *a*, and the localization of window can be translated by translating parameter *τ*.

The main difference between DWT and CWT is that the scaling and translating parameters of DWT are discretized by power function.

In practice, DWT is often designed through multiresolution analysis. Multiresolution analysis is also called the Mallat algorithm [40]. The flow of the Mallat algorithm is as follows: select a wavelet first and extend and translate the mother wavelet to get a set of wavelets. The signal passes through a high-pass filter and a low-pass filter, followed by the downsampling process (dyadic decimation, that is, keep the even indexed elements), then the detail coefficients (cD) and the approximation coefficients (cA) are obtained. Next, the approximation coefficients replace the original signal and use the same scheme to decompose and so on.

Since the wavelet coefficients obtained by convolving with the signal at different resolutions are the representations of the original signal at different resolutions, that is, the wavelet coefficients reflect the frequency components of the heartbeat signals along the timeline. We use the approximation coefficients and the detail coefficients at the last layer of DWT as the time-frequency features of heartbeat signals.

Similarly, we also give an example to illustrate the validity of the wavelet coefficients features. We choose three heartbeat classes, namely, class A, class J, and class /. 50 samples are randomly chosen from each class. Then, we calculate the mean of the approximation coefficients and the detail coefficients of these samples, respectively.  Figure 4 shows that the extracted approximation coefficients and detail coefficients have obvious difference among these classes.

### 4.6. ELM for Heartbeat Classification

In the feature extraction stage, RR interval features and wavelet time-frequency features are extracted. Then, these features are concatenated as the inputs of ELM, as shown in Figure 5.

The number of the output nodes in ELM is set to be the same as the number of heartbeat classes. During the offline training phase, the original labels of the heartbeat training samples are encoded to the matrix form in equation 4 and the output parameters *β* are analytically calculated using equation 7^.^

During the online classification phase, when the heartbeat sample *x* comes and needs to be classified, the output vector of ELM to sample *x*, *f*(*x*)=[*f*_1_(*x*),…,*f*_*m*_(*x*)]^*T*^ with *f*_*j*_(*x*) being the output of the *j*th output node, is calculated by

(9) $$\begin{array}{c} f\left(x\right)=h\left(x\right)\beta , \end{array}$$

where *h*(*x*)=[*h*_1_(*x*),…, *h*_*L*_(*x*)] is the output vector of the hidden layer with respect to *x*.

Finally, the predicted class label of heartbeat sample *x* is

(10) $$\begin{array}{c} \text{label}\left(x\right)=\underset{j\in \left\{1,\ldots ,m\right\}}{\arg\max}f_{j}\left(x\right). \end{array}$$

### 4.7. Parameter Design

In our proposed approach, four parameters need to be preset, including the wavelet type of DWT, the number of decomposition layers of DWT, regularized parameter, and the number of hidden nodes in ELM. We first use the grid search method to determine the wavelet type and the number of decomposition layers according to the accuracy of validation set. Then, grid search is carried out again to select the combination of regularized parameter and the number of hidden nodes based on the accuracy on validation set.

## 5. Experimental Study

### 5.1. Dataset Division

In our experiments, 13% of the class N, 40% of the classes L, R, A, V, and P, and 50% of the remaining classes are randomly selected to constitute the training set. The remaining samples make up the testing set.  Table 2 gives the detailed dataset partition of the MIT-BIH arrhythmia dataset.

### 5.2. Performance Metrics

We evaluate classification performance in terms of the class sensitivity (Se), the class positive predictivity (Pp), and overall accuracy. The class sensitivity reflects the proportion of the samples with positive model predictions in these with positive true labels. The class positive predictivity denotes the proportion of the samples with positive true labels in all the samples with positive model predictions. They are calculated as follows:

(11) $$\begin{array}{c} \text{Se}=\frac{\text{TP}}{\text{TP}+\text{FN}}\times 100\%, \end{array}$$

(12) $$\begin{array}{c} Pp=\frac{\text{TP}}{\text{TP}+\text{FP}}\times 100\%, \end{array}$$

(13) $$\begin{array}{c} \text{Acc}=\frac{\text{TP }+\text{ TN}}{\text{TP }+\text{ TN }+\text{ FP }+\text{ FN}}\times 100\%. \end{array}$$

where TP, TN, FN, and FP are the number of true positives, true negatives, false negatives, and false positives, respectively.

### 5.3. User-Specified Parameters

In our experiments, we first standardize the extracted features by

(14) $$\begin{array}{c} x^{*}=\frac{x-\mu }{\sigma }, \end{array}$$

where *μ* and *σ* are the mean and standard deviation of features. The standardized data satisfy the mean value of 0 and the variance of 1.

The wavelet type and the number of decomposition layers need to be carefully designed for DWT. Many types of wavelets can be used for DWT. These wavelets have different waveforms and lengths. The number of wavelet decomposition layers affects the decomposition granularity of heartbeat signals. We conduct experiments to study the influence of different wavelet types and the number of wavelet decomposition layers on heartbeat classification. The number of layers that a wavelet can be decomposed is related to the frequency of the original signal, so the number of decomposition levels of some wavelets is limited. In our experiments, we select four typical types of wavelet families, namely, Daubechies wavelets, Biorthogonal wavelets, ReverseBior wavelets, and Symlets wavelets. Then, we select a representative wavelet from each wavelet family, respectively. The number of decomposition layers ranges from 2 to 6. In the experiment, we set the number of hidden layer nodes of ELM to 3000, and the regularization parameter to 0.1.  Table 3 shows the experimental results. Db1 with 5-level decomposition achieves the highest accuracy. For db1, bior1.3, and sym2 wavelets, 5-level decomposition has the highest accuracy. For the rbio3.1 wavelet, the classification accuracies of 3-level, 4-level, and 5-level are similar. The higher the number of wavelet decomposition levels, the smaller the number of wavelet coefficients at the highest layer. In our proposed approach, wavelet approximation coefficients and detail coefficients of the highest layer are adopted as the features of the heartbeat signal. A smaller number of features can reduce the complexity and classification time. Therefore, 5-layer decomposition is suitable.  Table 3 also gives the total number of the approximation coefficients and detail coefficients at each decomposition layer.

In ELM, the regularization parameter *C* and the number of hidden layer nodes *L* are two key parameters that affect the classification performance. The optimal combination of *C* and *L* for ELM is determined by the accuracy on validation set in our experiment. The ranges of grid search for *C* and *L* are {10^−4^, 10^−3^,…, 10^4^, 10^5^} and {200,400,…, 5000}, respectively. The activation function uses sigmoid function. The parameters of sigmoid function are randomly generated within [−1, 1] based on uniform distribution.  Figure 6 shows the results of grid search on validation set. We observe that a smaller number of hidden nodes cannot obtain good classification accuracy. When the number of hidden layer nodes reaches 3000, continuing to increase *L* will not produce greater gains. For regularized parameter *C*, a value of 0.1 or 1 is appropriate for heartbeat classification.

### 5.4. Experimental Results

We compare the proposed algorithm with four classic classification algorithms, including BPNN, KNN, SVM, and decision tree (DT). RR interval features and wavelet coefficients features are extracted as the features of heartbeat signals. Daubechies 1 is used, and DWT performs 5-layer wavelet decomposition. The approximation and detail coefficients at the fifth layer are served as the wavelet features of heartbeat signals. In the training samples, 70% are used for training the classifier and 30% are used as the validation set. According to the accuracy on the validation set, the hyperparameters of the classifier are determined. The number of the hidden layer neurons of BPNN is consistent with that of ELM for comparison. And the parameters of BPNN are trained using stochastic gradient descent (SGD), which runs iteratively. SVM cannot achieve multiclassification task. One-against-one (OAO) strategy is used to extend SVM to multiclassification. In our experiment, 16 types of heartbeats need to be classified, so the number of SVMs required is 16*∗*15/2 = 120. The comparison results are shown in Table 4. We can find that ELM achieves the highest accuracy, the decision tree has the lowest, and the performance of KNN and SVM is comparable.

Table 5 shows the sensitivity and positive predictability of each heartbeat class. Most of the classes present satisfactory classification performance, except for the classes a, J, e, and Q. In addition, Table 6 gives the confusion matrix of the heartbeat classification, from which we can observe the detailed classification results. Totally, 27 samples are misclassified for class a, of which 10 samples are misclassified as N, 11 are misclassified as A, and 4 are misclassified as V. The reason is that class a has no significant morphological differences compared with the other three misclassified classes. Similarly, 26 samples for class J are misclassified, of which 22 samples are misclassified as N.

The strong morphology similarity between classes J and N in record 234 may be responsible for the misclassifications. All samples are misclassified in all 8 samples of class e. This is because in record 223, the morphological differences between classes e and N are hardly observed. All the samples of class Q are misclassified. We observe from the ECG of class Q that its waveform appears as irregular and large-amplitude fluctuation. The cardiovascular experts label these samples as unclassified samples, so how to reduce the signal deformation and loss of these samples is the key issue, but this is beyond the scope of our study.

We also compare the training time and testing time of different classifiers. The results are shown in Table 7. The training time of BPNN is quite time-consuming. Although DT shows the least training and testing time, it does not reach a satisfactory classification accuracy as shown in Table 4. The total time of ELM training and testing time is less than that of SVM and KNN, which shows the efficiency of the ELM algorithm.

## 6. Conclusions

In this paper, we propose an efficient ELM approach for automatic heartbeat classification. We extract the temporal features and wavelet time-frequency features for heartbeat signals. Four RR intervals are calculated in time domain, which reflects the dynamic information of heartbeat signals. We also employ DWT to decompose each heartbeat signal. We use the detail coefficients and approximation coefficients at the fifth level, a total of 16 wavelet coefficients, as the time-frequency features for the heartbeat signals. The ELM algorithm is developed for multiclass heartbeat classification. Experimental results using the MIT-BIH arrhythmia dataset show that our proposed approach achieves better recognition accuracy and less computational time in comparison with existing classification approaches. Besides, we give a reference for choosing the wavelet and the number of wavelet decomposition levels of DWT, which is instructive for employing DWT as a feature extractor in automatic heartbeat classification. However, due to the random assignment of the hidden layer parameters in ELM, the classification accuracy may fluctuate. As the future work, ensemble learning can be considered in the ELM-based heartbeat classification approach to increase the classification accuracy and stability. In addition, the multilayer structure with multiple hidden layers can be studied for ELM to enhance the heartbeat signal classification performance.

## Figures and Tables

**Figure 1:** The structure of ELM.

**Figure 2:** The overall structure of the proposed approach.

**Figure 3:** Examples of the distributions of four RR intervals for different heartbeat classes.

**Figure 4:** Example of the wavelet coefficient features extracted for different heartbeat classes. (a) The approximation coefficients. (b) The detail coefficients.

**Figure 5:** Schematic diagram of the proposed ELM approach for heartbeat classification.

**Figure 6:** Accuracies of different combinations of *C* and *L* on validation set.

**Table 1:** The detailed description of the MIT-BIH arrhythmia dataset.

Heartbeat type	Abbreviation	Annotation
Normal beat	NOR	N
Left bundle branch block	LBBB	L
Right bundle branch block	RBBB	R
Atrial premature contraction	APC	A
Premature ventricular contraction	PVC	V
Paced beat	PACE	/
Aberrated atrial premature beat	AP	a
Ventricular flutter wave	VF	!
Fusion of ventricular and normal beat	VFN	F
Blocked atrial premature beat	BAP	x
Nodal (junctional) escape beat	NE	j
Fusion of paced and normal beat	FPN	f
Ventricular escape beat	VE	E
Nodal (junctional) premature beat	NP	J
Atrial escape beat	AE	e
Unclassifiable beat	UN	Q
Total	—	16

**Table 2:** Training set and testing set division of the MIT-BIH arrhythmia dataset.

Heartbeat type	Total	Training	Testing
Normal beat	75023	9753	65270
Left bundle branch block	8072	3229	4843
Right bundle branch block	7255	2902	4353
Atrial premature contraction	2546	1018	1528
Premature ventricular contraction	7129	2852	4277
Paced beat	7026	2810	4216
Aberrated atrial premature beat	150	75	75
Ventricular flutter wave	472	236	236
Fusion of ventricular and normal beat	802	401	401
Blocked atrial premature beat	193	96	97
Nodal (junctional) escape beat	229	114	115
Fusion of paced and normal beat	982	491	491
Ventricular escape beat	106	53	53
Nodal (junctional) premature beat	83	42	41
Atrial escape beat	16	8	8
Unclassifiable beat	33	16	17
Total	110117	24096	86021

**Table 3:** Results of different wavelets and decomposition levels.

Wavelet	Decomposition level	The number of wavelet coefficients	Accuracy (%)
db1	2	118	97.12
	3	60	97.88
	4	30	98.39
	5	16	98.43
	6	8	97.55

bior1.3	2	124	97.18
	3	66	97.60
	4	38	97.94
	5	24	98.21
	6	—	—

rbio3.1	2	120	97.81
	3	62	98.22
	4	34	98.26
	5	20	98.24
	6	12	97.28

sym2	2	120	96.28
	3	62	97.01
	4	34	97.94
	5	20	98.25
	6	12	97.68

**Table 4:** The comparison results with other approaches.

Features	Classifier	Accuracy (%)
RR + db1 (5-level)	BPNN	97.71
	KNN	98.31
	SVM (OVO)	98.38
	DT	95.84
	ELM	98.61

**Table 5:** Sensitivity and positive predictivity for each heartbeat class.

Heartbeat type	Test	Se (%)	Pp (%)
N	65270	99.28	99.35
L	4843	99.40	99.03
R	4353	99.22	98.58
A	1528	88.81	87.27
V	4277	95.25	95.63
/	4216	99.79	99.03
a	75	64.00	77.42
!	236	91.95	93.53
F	401	83.04	79.47
x	97	86.46	97.65
j	115	73.68	61.31
f	491	86.35	87.78
E	53	92.45	100.00
J	41	36.59	88.24
e	8	0.00	0.00
Q	17	0.00	0.00
Total	86021	98.61	98.61

**Table 6:** Confusion matrix.

	Predict labels																
		N	L	R	A	V	/	a	!	F	x	j	f	E	J	e	Q
True labels	N	64803	20	47	128	129	1	4	14	36	1	51	35	0	1	0	0
	L	14	4812	1	1	9	1	0	0	0	0	0	5	0	0	0	0
	R	20	0	4319	11	2	0	0	0	0	0	0	0	0	1	0	0
	A	143	4	1	1357	11	1	6	0	0	1	1	2	0	0	1	0
	V	85	16	3	33	4074	4	4	1	49	0	0	8	0	0	0	0
	/	4	1	0	0	0	4207	0	0	0	0	0	4	0	0	0	0
	a	10	0	0	11	4	1	48	0	0	0	0	1	0	0	0	0
	!	9	0	0	1	7	1	0	217	0	0	0	1	0	0	0	0
	F	42	2	2	2	20	0	0	0	333	0	0	0	0	0	0	0
	x	5	0	0	6	2	0	0	0	0	83	0	0	0	0	0	0
	j	21	0	5	3	0	0	0	0	0	0	84	1	0	0	0	0
	f	33	2	0	0	0	32	0	0	0	0	0	424	0	0	0	0
	E	2	0	1	0	0	0	0	0	0	0	1	0	49	0	0	0
	J	22	0	2	2	0	0	0	0	0	0	0	0	0	15	0	0
	e	8	0	0	0	0	0	0	0	0	0	0	0	0	0	0	0
	Q	9	2	0	0	2	0	0	0	1	0	0	2	0	0	0	0

**Table 7:** Comparison of running speeds of different classifiers.

Classifier	Training time (s)	Testing time (s)	Total time (s)
BPNN	655.02	6.88	661.9
KNN	0.16	17.92	18.08
SVM (OVO)	5.01	16.83	21.84
DT	0.76	0.03	0.79
ELM	9.17	8.25	17.42

## Data Availability

The data used to support the findings of this study are included within the article.
